# Kinematic Diagnosis of Throwing Motion of the Chinese Elite Female Discus Athletes Who Are Preparing for the Tokyo Olympic Games

**DOI:** 10.1155/2022/3334225

**Published:** 2022-09-22

**Authors:** Lixia Wang, Lina Hao, Bo Zhang

**Affiliations:** ^1^Capital University of Physical Education and Sport, Graduate Student Department, Beijing 100191, China; ^2^Sport College of Shijiazhuang University, Shijiazhuang, 050035 Hebei, China; ^3^Hebei Medical University, Shijiazhuang, 050017 Hebei, China; ^4^The Tian Jia Bing Middle School Attached to Hebei Normal University, Shijiazhuang, 050035 Hebei, China

## Abstract

The purpose of this study was to examine the difference of kinematic skill characteristics between the Chinese and world elite female discus athletes. We used the methods of literature, three-dimensional video analysis, and mathematical statistics to compare and analyze the differences of some kinematic parameters between the three Chinese female discus athletes and four world female discus athletes. The result shows that the speed of discus release of the Chinese elite female discus athletes is lower (*p* < 0.05) than that of the world elite female discus athletes. Compared to the world elite female discus athletes, the height of release is higher (*p* < 0.05). But there was no significant difference in the angle of release (*p* > 0.05), rotation rhythm (*p* > 0.05), and discus speed increment (*p* > 0.05) in different stages during the throwing procedure from double support stage to delivery stage. The results may provide reference for the special technique training of the Chinese female discus throwers, so as to improve the discus throwing level of Chinese women.

## 1. Introduction

Discus throwing is one of the four throwing events in track and field. Female discus throwing is the first throwing event to reach the world top level in the history of Chinese track and field. It is a sport event which needs to achieve the highest release speed and the longest throwing distance. Therefore, discus athletes need to possess certain physical strength and special kinematic skills [1] to complete the complex movements in the restricted area at high speed [2–4]. During the procedure of discus throwing, it mainly includes three technical stages: holding the discus and preswing, rotation, and delivery, maintaining body balance after releasing the discus [5]. In different stages, throwers must control the motion in precise kinematic skills. And the discus throwing skills are constantly changing to improve the throwing performance. In the 1970s, the introduction of wide standing, low posture, and wide back rotating throwing techniques, which are popular in the world, has greatly promoted the development of women's discus throwing in China. Chen Yang, Feng Bin, and Su Xinyue as the leading figures in Chinese female discus athletes have promoted and led the development of Chinese female discus throw. Although the three Chinese elite female discus athletes have achieved excellent sports performance, there is still a certain gap with the world elite female discus athletes. How to improve the throwing performance of the Chinese elite female discus athletes has become an important subject of current research.

## 2. Literature Review

Many researchers analyzed the factors that determined the throwing performance from multiple perspectives. Takanashi et al. study the relation between the competitive performance and athlete maximum lifting weighting [6]. In order to carry out special strength training targeted, Dinu et al. analyzed the muscle activation patterns during the discus throwing process [7]. More research focuses on the kinematic diagnosis of discus throwing.

Performance in discus throw mainly depends on the maximum speed, optimum height, and specific angle of the discus at release [1, 2, 7, 8]; the speed and angle of the discus release are not independent but affect each other [9]. These two factors are important to the performance. Especially the release speed of discus is the most critical variable in achieving high-level athletic performance [1, 2, 4, 10–15]. It also has been mentioned in some literatures that the correlation coefficient between release speed and official throwing distance is 0.8657 [16]. In order to improve vertical and horizontal release speed, female discus athletes use more complex techniques than male discus athletes [11]. It has been pointed that if release speed increases from 24.5 m/s to 25.5 m/s, the throwing performance will be improved by 4.8 m [17]. The release speed of the world's top athletes ranges from 22 to 25.5 m/s, which is also the speed level required to achieve the result of more than 60 m [18]. About the angle of release, some study has pointed out that the reasonable release angle depends on the velocity and direction of wind and athletes' physical conditions [19]. The increase of discus release angle may reduce the release speed. Elite discus athletes have a personalized optimal release angle. Some studies believe that the angle of release is usually between 25° and 40° [20]. Regarding the release height, different study put forward different suggestions. Early study found that the release height of elite women discus throwers was 1.48 m [21]. In another study, it is put forward that the optimum height of release is 90% of thrower's height [22], while Bartlett think that 93% of thrower's height is the best release height. Of course, in addition to technical parameters, there are anthropometric indicators such as athlete's height and arm length of athletes [1]; other studies also indicate that the height of release is important to performance of discus throwing [23, 24].

The time in each stage of rotary discus throwing can reflect the rhythm and performance, which is an important technical characteristic of excellent rotary discus throw athletes [25]. The discus throw technique is a process in which the moving human body drives the discus to rotate and accelerate [26, 27]. The change of center of body gravity and discus speed in the whole process of discus throwing can also be used to judge the quality of athletes' rotating skills [28, 29].

Few studies have researched the kinematic difference between the three top Chinese discus athletes and world elite female discus athletes. The purpose of present study was to compare the kinematic difference and find the shortcoming in throwing action of the three Chinese elite female discus athletes. It was hypothesized that discus release parameters, rotation rhythm, and discus speed increment in each stage of the three Chinese elite discus athletes would be significantly different compared to the world elite female throwers. The significance of this research is to provide a reference for the special technical training of the three Chinese female discus athletes who are preparing for the Tokyo Olympic Games, so as to improve the level of Chinese female discus.

## 3. Research Methodology

### 3.1. Participants

This study tested the three Chinese elite female discus athletes who are preparing for the Tokyo Olympic Games. The basic information of the three Chinese elite female discus athletes (right-handed discus athletes) can be seen in Table 1. They were Chen Yang, Feng Bing, and Su Xinyue (Chen, Feng, and Su for short) who were the three top discus athletes of the national team of China. This study was approved by the Ethics Committee of Capital University of Physical Education and Sport. All the throwers were informed of the purpose of the research and signed a consent form before participating. Data of the four world elite female discus (Perkovic who won the 2011 IAAF Diamond League champion in Shanghai and the top three female discus athletes in 1993 IAAF World Championships) were obtained from documents; the availability of these data has been proven in research [28, 29]. The basic information about these athletes can be seen in Table 2.

### 3.2. Three-Dimensional Video Recording and Motion Analysis

After finishing the discus throwing-specific warming up, throwers went to the outdoor discus throwing area, and each thrower performed six maximal effort throwing instructed according to the criteria of IAAF. The interval time between two throws for each thrower was as long as the player feels ready to start the next throw. And we choose the two best performances of six throws of each athlete as the study data (Table 2). In this study, each throw of every athlete was recorded by using three digitals' camcorders (Panasonic GH5S, 100 Hz). Two Panasonic GH5S high-speed camcorders were located behind the throw circle and on the right side of the discus throw circle, respectively, with a 90° angle between two camcorders (Figure 1). Both distance were 10 meters far from the center of discus throw circle. The height of camcorder was 1.2 m. A calibration frame (2018 QF-28: 2 m × 2 m × 2.5 m) with 28 calibration points was set out at the throw circle and used for spatial reference. The camera was turned on before the first throwing and not turned off in the middle for continuous shooting to record the throwing movements. For being convenient to analysis, in this study, each throw (take the right hand throwing for example) was divided into five consecutive phases by six critical moment (Figure 2): (1) the maximum preswing; (2) the right foot off the ground (R↑); (3) the left foot off the ground (L↑); (4) the right foot touches the ground (R↓); (5) the left foot touches the ground (L↓); and (6) discus release (♂). The five consecutive phases in sequence are the following: (A) double support stage (maximum preswing to R↑); (B) single support stage (R↑ to L↑); (C) airborne stage (L↑ to R↓); (D) transition stage (R↓ to L↓); and (E) delivery stage (L↓ to ♂) [2–4, 7].

### 3.3. Three-Dimensional Kinematic Data Processing

Signal TEC3D-Video (3D Video parsing software 2.0 Chinese Version) was used to parse the digital video. The comprehensive average error and maximum error of 3D calibration are less than 0.05. Choose the Japanese-M model with center of human body gravity (21points, 16 links), and add a discus center point. In the video clip process, the method is as follow: each throw video clip of the two camcorders was digitized from the first 5 frames at the end of the maximum backswing to 4 frames after the discus release [4, 11]. Time synchronization of 2D video coordinate data of two VCRS by using multikeyframe method [2] used DHL method to synthesize time-synchronized 2D coordinate data into 3D coordinate data.

The cubic spline data interpolation method is adopted, and the optimal low-pass filter (0.16) is used for digital filtering to smooth the original data. The filtering truncation frequency is 8 Hz. After automatic data calculation and processing (interpolation and filtering of original coordinates, filtering of transformed coordinates, etc.), the calculated results are filtered.

### 3.4. Statistical Analysis

IBM SPSS20.0 software was used to conduct independent sample *t*-test, and the statistical significance of this study was defined as a class I error probability not greater than 0.05 (*p* < 0.05).

## 4. Results

### 4.1. Comparison of Performance Variables

Vacuum flight distance refers to the theoretical flight distance of discus after removing the influence of fluid, which is calculated by the following formula [2]:

(1) $$\begin{array}{c} \text{d}=\frac{\left\{{S_{R}}^{2}\sin\theta_{R}\cos\theta_{R}+S_{R}\cos\theta_{R}\sqrt{\left[{\left(S_{R}\sin\theta_{R}\right)}^{2}+2gh_{R}\right.}\right\}}{\text{g}}, \end{array}$$

where *S*_*R*_ is release speed, *h*_*R*_ is release height, and *θ*_R_ is release angle (*g* = 9.80 m/s^2^).

Aerodynamic distance is the difference between throwing performance and vacuum flight distance. Discus throw performance is the sum of vacuum flight distance, aerodynamic distance, and release loss distance [1, 2]. Vacuum flight distance is the main component of official throwing distance.

The average throwing performance (60.90 ± 3.60 m) and vacuum flight distance (54.12 ± 2.30 m) of the three Chinese elite female discus athletes were significantly lower (*p* < 0.05) than that of the four world elite female discus athletes (65.90 ± 1.01 m and 59.92 ± 2.18 m), while the aerodynamic distance has no significant difference (*p* > 0.05) between the Chinese and world elite female discus athletes (Table 3).

### 4.2. Comparison of Discus Release Parameters

In this study (Table 4), the mean discus release speed of the three Chinese female discus athletes (23.10 ± 0.56 m.s^−1^) was significantly lower (*p* < 0.05) than that of the world elite female discus athletes (24.37 ± 0.33 m.s^−1^). The mean discus release height (1.63 ± 0.34 m) was significantly higher (*p* < 0.05) than that of the world elite female discus athletes (1.52 ± 0.43 m), but it was lower than 1.65 meters. The difference of release angle (36.52 ± 1.53° vs. 36.85 ± 2.73° of the Chinese and world elite female discus athletes, respectively) was not significant (*p* > 0.05).

### 4.3. Comparison of Rotation Rhythm

In this study (Figure 3), Feng's total time spent in each throwing action was the longest, and the mean time Feng spent in two throwing procedure was 1.49 s; Chen's mean time spent in two throwing procedure was the shortest (1.27 s) of all throwers; and Su's mean time spent in two throwing procedure was 1.28 s shorter than that of the four world elite female discus athletes (1.32 s) too.

The mean time percentage spent in each stage of the three top Chinese and four world elite female discus athletes was 38.83% vs. 33.00% (double support stage), 30.33% vs. 33.75% (single support stage), 6.83% vs. 7.25% (airborne stage), 11.33% vs. 13.00 (transition stage), and 12.67% vs. 13.00% (delivery stage), respectively.

From Table 5, we found that, compared with the four world elite female discus athletes, the mean time spent in double support stage of the three top Chinese female athletes was significantly long (*p* < 0.05), but there were no significant difference in other four stage of throwing action (*p* > 0.05).

The mean time spent in full throwing action of the three top Chinese female discus athletes (1.35 s ± 0.11) compared with the four world elite female discus athletes (1.32 s ± 0.01) had no significant difference (*p* = 0.544).

### 4.4. Comparison of Discus Speed Increment in Each Stage

In this study, we found that the average discus speed of the three Chinese elite female discus athletes showed a nearly upward trend from the moment of maximum preswing to the discus release. Especially during the delivery stage, the speed of discus increased quickly and largely. It is a little drop in the moment of right foot touching ground compared to the moment of left foot landed. The average speed of the center of body gravity showed an upward trend from the moment of maximum preswing to the right foot touching ground. And then at the moment of left foot touching ground, the velocity of the center of body gravity was lower than that of the right foot touching ground and continues to decrease until discus release (Figure 4).

As can be seen in Table 6, during the double support stage, the average increment of discus speed of the three Chinese elite female discus athletes (4.08 ± 0.80 m.s^−1^) was greater than that of the four world elite female discus athletes (1.70 ± 0.76 m.s^−1^); it has a significant difference (*p* < 0.05).

During the single support stage, the average increment of discus speed (3.97 ± 1.58 m.s^−1^ vs. 4.72 ± 0.68 m.s^−1^ by the Chinese and world elite female discus athletes, respectively) has no significant difference (*p* > 0.05).

During the airborne stage, the mean discus speed increment of the three Chinese elite female athletes was descend (−0.37 ± 2.20 m.s^−1^) while that of the four world elite female discus athletes was enhanced slightly (0.27 ± 1.59 m.s^−1^); it had no significance too (*p* = 0.671).

During transition stage, the average increment of discus speed was 2.47 ± 2.77 m.s^−1^ and 3.40 ± 1.07 m.s^−1^ by the Chinese and world elite female discus athletes, respectively. During delivery stage 12.32 ± 2.41 m.s^−1^ and 13.78 ± 2.11 m.s^−1^, respectively, both transition stage and delivery stage had no significant difference too (*p* = 0.602 vs. *p* = 0.403 by the Chinese and world elite female discus athletes, respectively), but we found that in transition stage and delivery stage, the discus speed increment of the three Chinese elite female discus athletes is less than that of the world elite female discus athletes.

## 5. Discussion

The purpose of this study was to examine the difference of kinematic skill characteristics between the Chinese elite female discus athletes and worlds'. Then, look for the shortcoming of the three Chinese elite female discus athletes who are preparing for the Tokyo Olympic Games. It was hypothesized that the release parameters, rotation rhythm, and discus speed's increment of the three Chinese elite female discus athletes who are preparing for the Tokyo Olympic Games is significantly different from those of the world elite female discus athletes.

### 5.1. Difference in Performance Variables

The results from the present study showed that the mean throwing performance of the Chinese and world elite female throwers had significant difference. The difference of vacuum flight distance as the main component of official throwing distance is also significant. But the aerodynamic distance had no significant difference (Table 3). These results suggest that we can improve the throwing performance from the aspects which affect the vacuum distance.

Discus athletes must carefully control their release parameters so that the discus is thrown at the maximum height, combined with optimal release angles, and maximum speed which is the most important factor contributing to the vacuum flight distance, and therefore long throws [1, 2].

### 5.2. Difference in Parameters of Discus Release

The results from the present study also showed that the height and speed of discus release had significant difference in the Chinese and world elite female discus athletes, although there was no obvious difference in the angles of discus release (Table 4). These results suggest that changes in throwing performance can be explained by main techniques combination. To improve the throwing performance, the Chinese elite female throwers should enhance the speed of discus release based on the maximum height and optimal angle of discus release, thus largely partly accepting the initial hypothesis. The Chinese elite female throwers may try to strengthen special strength training to improve speed of discus release, especially the muscles (LD, DM, and TM) that have constant activation during the whole movement [7]. Besides, limiting the variability of kinematics and muscular pattern has been associated with a better efficiency in discus throwing [8]. It is necessary to study the muscle activation patterns of the Chinese elite female discus throwers.

### 5.3. Difference in the Rhythm of Rotation

The results from the present study showed that there was no significant difference in the mean time spent in the whole throwing procedure between the Chinese and world elite female discus athletes (Table 5). But Feng's is significantly higher than the others (Figure 2). The results also showed that the mean time spent in double support stage of the three Chinese elite female discus athletes was significantly longer than that of the world's (Table 5). But there was no significant difference in single support stage, airborne stage, transition stage, and delivery stage (Table 5), thus largely partly rejecting the initial hypothesis.

Discus throwing action of each stage has different effect on the throwing performance [3, 8]. The techniques of double support stage require a stable center of gravity, which is of great significance to the formation of the whole rotation rhythm [30]. In this study three Chinese elite female discus athletes in accordance with the law that time spent in double support stage should be the longest [31]. Throwers should increase the distance between two feet and control the route of swinging legs in the single support stage and the individual's technical rhythm [32].

As reported in other study, the time spent in single support stage of the world elite athletes is about 0.40 s, accounting for about 32% of the total time [31]. The airborne stage is the deceleration stage of “body-discus” system [33]. In order to reduce the loss of horizontal velocity, this stage is short with small fluctuation of body gravity center [34]. Some studies point out that the time of the world elite male and female discus athletes in the airborne stage should be 0.1-0.2 s, accounting for 10%-15% of the total time [31].

About the time spent in transition stage having different ideas, if the time is too short and the landing speed is accelerated, the landing distance is bound to be short and the remaining range of discus is small, which further affects the effect of surpassing the equipment. If the time is too long, it will increase the amplitude of the discus and increase the difficulty of moving the upper limb to the left leg.

A study has pointed out that the time spent in the delivery stage of the world elite athletes is within the range of 0. 10-0. 20 s [35]; Viitasalo et al. proposed that the time spend in transition phase (49.5%) and delivery phase (50.5%) is basically equal, which is helpful for athletes to obtain the optimal conditions of delivery in transition phase, thus producing higher release speed [9].

This study suggest that the Chinese elite discus athletes should maintain and improve the better rotation rhythm according to personal technical characteristics.

### 5.4. Difference in Discus Speed Increment at Each Stage during Throwing Process

The result from this study showed that the speed of discus of the three Chinese elite female discus athletes showed nearly an upward trend during the whole throwing process. The speed of body center of gravity increased first and then decreased (Figure 4). The result suggests that during the throwing process, the movement of discus throwers follows the biomechanical principle of discus throwing basically.

But the result from present study also showed that the mean increment of the discus speed of the three Chinese female discus athletes was significantly higher than that of the world's in double support stage (Table 6). The result suggest that the three Chinese elite female discus athletes are eager to accelerate in the double support stage, and the speed increases too fast, which is easy to destroy the overall rhythm of rotation and is not conducive to the play of subsequent movements.

From the result of this study, there were no significant difference in other four stage (single support stage, transition stage, airborne stage, and delivery stage), but the mean increment of discus speed of the three Chinese elite female discus athletes is all lower than that of the worlds' (Table 6). Especially in the airborne stage, the discus speed increment of the world elite female discus athletes was positive value, but the three Chinese elite female discus athletes were negative value, thus partly rejecting the initial hypothesis.

The result suggest that the three Chinese elite female discus athletes should increase the discus speed increment in single support stage, airborne stage, transition stage, and delivery stage, in order to increase the speed of release. But in different stage, the discus speed should keep changing. In order to form the position of body leading beyond the discus, in the airborne stage, the speed of discus will be down, until the left foot touches the ground [35], but the discus speed increment should be positive value.

The delivery stage with the largest increment of discus speed and the largest contribution rate to discus release speed is the most important technical link to determine the throwing distance. Unless in the double support stage, the three Chinese elite female discus athletes should increase the discus speed increment in each stage from the perspective of rotating skills and specific strength training. According to the individual technical characteristics of athletes, the rhythm of the rotation technique should be further improved. In addition, according to the muscle activation characteristics of the main muscle groups that affect the discus performance, explosive strength training should be carried out for the muscle groups that contribute a lot to the discus performance.

### 5.5. Research Limitation

In this study, we only collected partly 3D kinematic parameters of discus throw techniques of the four world elite female discus athletes, such as release speed, angle and height of release, rotation rhythm, and discus speed increment in different movement stages. While the hip-shoulder and shoulder-arm separation angles and trunk forward-backward tilt angle which also have an important impact on performance in discus throw have not been collected, it is hoped that in the future, we can collect the 3D kinematic parameters of the world and Chinese elite female discus athletes in the same competition for a comprehensive comparative analysis.

## 6. Conclusion

The result of this study indicates the difference of discus release parameters in Chinese and world elite female discus throwers. We found that the lower release speed is the key to restrict the Chinese elite female discus athletes to achieve the excellent performance. The result suggests that three Chinese elite female discus athletes should aim to increase the speed of discus release. The result of this study also indicates slight similarity and difference in the rotation rhythm and discus speed increment. The rotation rhythm has similarity and personality characteristics. During the whole throwing, in addition to the double support stage, the increment of discus speed is lower than that of the world elite female discus athletes in other four stage, although there was no significant difference. The result also suggests that Chinese elite female discus athletes should improve the rotation technique and special strength training.

## Figures and Tables

**Figure 1:** 3D kinematic shooting diagram.

**Figure 2:** Diagram of discus throwing stage division.

**Figure 3:** The time spent in each stage of throwing action and total.

**Figure 4:** Average speed of body center and discus of the three Chinese elite female discus athletes.

**Table 1:** Basic information of the three Chinese elite female discus athletes.

Name	Age (year)	Height (m)	Body weight (kg)	PB (m)
Chen Yang	31	1.8	97	67.03
Feng Bing	28	1.84	95	66
Su Xinyue	31	1.78	95	65.59
Mean ± S	30 ± 1.73	1.81 ± 0.02	95.67 ± 0.94	66.21 ± 0.61

**Table 2:** Basic information of the research objects and performance used for analysis.

	Name	Nationality	Research performance (m)	Grade
Chinese	Chen 1	China	65.85	Athlete
	Chen 2		65.13	
	Feng 1	China	59.37	Athlete
	Feng 2		58.89	
	Su 1	China	58.10	Athlete
	Su 2		58.05	

World	Sandra Perkovic	Croatia	65.58	Athlete
	Olga Burova	Russia	67.40	Athlete
	Daniela Costain	Australian	65.36	Athlete
	Min Chun Feng	China	65.26	Athlete

**Table 3:** Comparison of distance variables between the Chinese and world elite female discus athletes.

Parameters	Chinese elite female discus thrower (*n* = 6)	World elite female discus thrower (*n* = 4)	*t*	*p*
Throwing performance (m)	60.90 ± 3.60	65.90 ± 1.01	-3.22	0.018^∗^
Vacuum flight distance (m)	54.12 ± 2.30	59.92 ± 2.18	-3.977	0.004^∗^
Aerodynamic distance (m)	6.78 ± 2.13	5.98 ± 2.44	0.548	0.599

**Table 4:** Comparison of discus release parameters between the Chinese and world elite female discus athletes.

Parameters	Chinese elite female discus thrower (*n* = 6)	World elite female discus thrower (*n* = 4)	*t*	*p*
Release angle (°)	36.52 ± 1.53	36.85 ± 2.73	-0.253	0.806
Release height (m)	1.63 ± 0.34	1.52 ± 0.43	4.694	0.002^∗^
Release speed (m.s^−1^)	23.10 ± 0.56	24.37 ± 0.33	-4.034	0.004^∗^

**Table 5:** Comparison of throwing time between the Chinese and world elite female discus athletes (s).

Movement phases	Chinese elite female discus athletes (*n* = 6)	World elite female discus athletes (*n* = 4)	*t*	*p*
Double support stage	0.52 ± 0.06	0.44 ± 0.03	2.528	0.035 ∗
Single support stage	0.41 ± 0.03	0.44 ± 0.04	-1.636	0.14
Airborne stage	0.09 ± 0.01	0.09 ± 0.02	-0.087	0.933
Transition stage	0.15 ± 0.03	0.17 ± 0.04	-0.954	0.368
Delivery stage	0.17 ± 0.04	0.13 ± 0.09	0.988	0.352
Total time	1.35 ± 0.11	1.32 ± 0.01	0.649	0.544

**Table 6:** Comparison of discus speed increment of the Chinese and world elite female discus athletes (m.s^−1^).

Movement phases	Chinese elite female discus thrower (*n* = 6)	World elite female discus thrower (*n* = 4)	*t*	*p*
Double support stage	4.08 ± 0.80	1.70 ± 0.76	4.263	0.004^∗^
Single support stage	3.97 ± 1.58	4.72 ± 0.68	-1.006	0.348
Airborne stage	−0.37 ± 2.20	0.27 ± 1.59	-0.443	0.671
Transition stage	2.47 ± 2.77	3.40 ± 1.07	-0.547	0.602
Delivery stage	12.32 ± 2.41	13.78 ± 2.11	-0.889	0.403

## Data Availability

The experimental data used and analyzed to support the findings of this study are available from the corresponding author on reasonable request.
